# Deep Learning-Based Magnetic Resonance Imaging Image Features for Diagnosis of Anterior Cruciate Ligament Injury

**DOI:** 10.1155/2021/4076175

**Published:** 2021-07-02

**Authors:** Zijian Li, Shiyou Ren, Ri Zhou, Xiaocheng Jiang, Tian You, Canfeng Li, Wentao Zhang

**Affiliations:** Department of Sports Medicine and Rehabilitation, Peking University Shenzhen Hospital, Shenzhen 518036, China

## Abstract

To study and explore the adoption value of magnetic resonance imaging (MRI) in the diagnosis of anterior cruciate ligament (ACL) injuries, a multimodal feature fusion model based on deep learning was proposed for MRI diagnosis. After the related performance of the proposed algorithm was evaluated, it was utilized in the diagnosis of knee joint injuries. Thirty patients with knee joint injuries who came to our hospital for treatment were selected, and all patients were diagnosed with MRI based on deep learning multimodal feature fusion model (MRI group) and arthroscopy (arthroscopy group). The results showed that deep learning-based MRI sagittal plane detection had a great advantage and a high accuracy of 96.28% in the prediction task of ACL tearing. The sensitivity, specificity, and accuracy of MRI in the diagnosis of ACL injury was 96.78%, 90.62%, and 92.17%, respectively, and there was no considerable difference in contrast to the results obtained through arthroscopy (*P* > 0.05). The positive rate of acute ACL patients with bone contusion and medial collateral ligament injury was substantially superior to that of chronic injury. Moreover, the incidence of chronic injury ACL injury with meniscus tear and cartilage injury was notably higher than that of acute injury, with remarkable differences (*P* < 0.05). In summary, MRI images based on deep learning improved the sensitivity, specificity, and accuracy of ACL injury diagnosis and can accurately determined the type of ACL injury. In addition, it can provide reference information for clinical treatment plan selection and surgery and can be applied and promoted in clinical diagnosis.

## 1. Introduction

The knee joint is a very important compound joint in the human body, which not only undertakes frequent and complex movements but also is the most important weight-bearing joint of the human body [1]. Therefore, knee injuries are inevitable in life. Most knee injuries are caused by high-intensity exercises, sports competitions, and falls from high altitudes. The most common knee injuries include anterior cruciate ligament (ACL) injury and meniscus injury, and the combination of the two injuries is also common. According to reports, the incidence of ACL injury with meniscus injury was more than 85%, which may cause joint swelling, pain, and movement inconvenience in patients, thus substantially affecting the life and work of patients [2, 3]. In the case of knee injury, timely and accurate assessment of ACL injury is helpful to select the best treatment plan and effectively evaluate the prognosis of patients. It is of great clinical significance for patients to recover the normal stability and normal motor function of knee joint and to avoid or reduce the secondary injury of other knee joint structures [4]. Clinically, complete tears and partial tears are often taken as the basis for judging ACL damage [5]. All in all, the early and correct diagnosis after ACL injury is of great significance for the choice of clinical treatment plan and prognosis [6, 7].

The commonly used methods for diagnosing ACL injury are roughly classified into three categories, clinical stability examinations, such as anterior drawer test and axis shift test, imaging examinations such as ultrasound diagnosis, CT diagnosis, and MRI diagnosis, and arthroscopy [8]. Ultrasound examination and CT examination require high operational experience of medical staff. Arthroscopic diagnosis is an effective standard for ACL injury, but the inspection method is limited to the case of trauma [9]. Therefore, clinical stability check is an important method for doctors to check ACL injury. Due to the good tissue resolution and high spatial resolution, MRI can not only objectively evaluate knee joint injuries but also evaluate knee joint injuries such as meniscus injuries and cartilage injuries [10].

Since MRI examinations show high clinical diagnosis accuracy of ACL tears and meniscus, knee MRI has become the first choice for the diagnosis of knee joint injuries in recent years. The deep learning approaches can automatically learn multilayer features, which are very suitable for the auxiliary diagnosis of medical images [11]. At present, deep learning approaches have surpassed traditional medical image analysis methods and have made great progress in the field of knee MRI. Mayo et al. [12] developed a fully automatic knee joint magnetic resonance cartilage damage detection system based on deep learning. The system consisted of two CNN networks. The first CNN network was utilized for the rapid segmentation of cartilage and bone, while the second CNN network evaluated the structural abnormalities of articular cartilage. The total accuracy of the experiment reached 98.37%. Therefore, the deep learning-based MRI cartilage injury detection system of the knee joint shows a high diagnostic accuracy, can quickly analyze images, significantly saves the diagnostic time, and improves the diagnostic efficiency. This diagnosis method is worthy of promotion and adoption.

In summary, the knee joint injury patients were taken as the research object in this research. MRI images of patients were optimized based on deep learning algorithms, which were then applied to the diagnosis of knee joint injury patients, and the adoption value of MRI image diagnosis in ACL injury was evaluated.

## 2. Materials and Methods

### 2.1. Research Objects and Grouping

Thirty patients with knee joint injuries diagnosed in our Hospital from May 2019 to March 2020 were selected as the research objects. All patients underwent MRI and the results were compared with those obtained by arthroscopy. There were 21 males and 9 females. The age range of the patients was 18–75 years, and the average age was (37.82 ± 5.18) years. The patients were rolled into two groups according to diagnosis methods. One group was MRI diagnose and the other group was arthroscopic diagnose, and they were compared within the groups. The experimental process had been approved by the ethics committee of the hospital, and all subjects included in the study had signed the informed consent forms.

Inclusion criteria: (i) clinical symptoms were joint pain, swelling, joint instability, etc.; (ii) physical examination methods (anterior drawer test, Lachman test, etc.) showed at least one positive sign; (iii) those who aged 18–75 years old.

Exclusion criteria: (i) patients with a previous history of knee joints, such as tuberculosis arthritis and rheumatoid arthritis; (ii) the patient's joints were found to have tumors or tumor-like lesions through examination; (iii) patients with a history of knee surgery; (iv) patients whose age was under 18.

### 2.2. MRI Examination

The patient's original image was sent to a postprocessing workstation. Three associate chief doctors with more than five years of experience in MRI diagnosis in the radiology department performed oblique coronal and cross-sectional multiplane recombination. The thickness was 0.4 mm, and there was no spacing between the layers. The three-dimensional reconstructed ACL and its surrounding structures were observed, and consensus was reached and recorded through consultation. At the same time, the MRI scan sequences (T2WI-SPAIR sagittal images, T2WI cross-sectional images, etc.) were observed and analyzed, and the corresponding diagnostic opinions were recorded. According to the characteristics, continuity, edge, shape, and signal of ACL damage, whether ACL was damaged and the extent of damage were judged. According to the comprehensive literature, MRI diagnostic criteria of ACL injury were established, and the MRI signs of ACL injury were classified into four categories [13] as follows. Grade 0: no abnormalities in initial profile, walk, and signal. Grade I: the ligament continuity was still good, the contour was still intact, the ligament was not thickened or slightly thickened and expanded, small patches or streaks of signal can be seen, and damage area was less than 50%. Grade II: ligamentous continuity was poor, but some continuous fibers were still visible; locally thickened or diffused ligaments were visible; incomplete or well-defined edges were at the site of ligament injury, or there were locally notched areas; abnormally high signal can be seen, with damage area greater than or equal to 50%. Grade III: there was intact rupture of the ligament, characterized by broken continuity of the ligament, displacement of the bent or broken end, clumpy ligament, increased signal, and unclear boundary.

After the patient's medical history and MRI results were provided, radiologists would observe and analyze the knee images of the patient to determine whether there was a tear in the ACL of the knee and the degree of the tear. If there was a difference of opinion, the three experts could reach a conclusion after consultation.

### 2.3. Arthroscopy Examination

Arthroscopy with a diameter of 4.0 mm and a wide angle of 30 degrees from Stryker and Smith & Nephew were utilized. The arthroscopy was performed by two joint surgeons. A detailed medical history was taken before surgery, and a physical examination was performed in combination with X-rays and MRI. The knee ACL was carefully examined during surgery. If there was a partial injury, a detailed examination with a probe was performed to avoid misdiagnosis. If a ligament injury was found arthroscopically, the physician could take further appropriate treatment and recorded the surgical plan and procedure. MRI findings and arthroscopic findings were studied and analyzed.

### 2.4. Deep Learning Model Construction Based on Multimodal Feature Fusion

#### 2.4.1. Deep Feature Extraction

At present, convolutional neural networks are more and more widely used in the field of medical image diagnosis and have made good progress. The mechanism of convolutional neural network refers to automatically performing the feature extraction of the image through the convolution operation of the image, and such feature has advanced semantic information and is more robust [14]. Since the deep learning model can only achieve ideal results when trained on annotated images, transfer learning is adopted to directly use the second to fifth convolution blocks of the pretrained VGG16 [15]. The feature map of the last layer of each convolution block is extracted, which is *H*(*g*), *g*=1,2,3,4,5. After the up-sampling *K*(*g* − 1) of *H*(*g* − 1) was obtained, the result image after 2^∗^2 convolution processing is pixel fused, and then, 5^∗^5 convolution kernel is used again to correct the fused image, which can eliminate the aliasing effect used above and obtain a new feature map *H*(*g* − 1). The pyramid fusion equation is as follows:

(1) $$\begin{array}{c} K\left(g-1\right)=y_{2\times 2}\left(H\left(g-1\right)\right),\\ H\left(g-1\right)=y_{5\times 5}\left(H\left(g\right)+H\left(g-1\right)\right). \end{array}$$

After the last layer *H*(2) is acquired, it passes through the batch normalization (BN) layer, the adaptive maximum pooling layer, and the fully connected layer in turn. The BN layer can speed up the convergence speed and classification effect of the model. *y*^(*n*)^ is set as the *n*th dimension feature of *H*(2), the BN layer is *H*(2) introduced with the parameters ∂^(*n*)^ and *D*^(*n*)^, and the indifference estimation is conducted to output the *n*th dimension feature as follows:

(2) $$\begin{array}{c} y^{\left(n\right)}=\partial^{\left(n\right)}{\bar{s}}^{\left(n\right)}+D^{\left(n\right)}, \end{array}$$

(3) $$\begin{array}{c} \bar{s_{l}}=\frac{s_{l}-q}{\sqrt{w_{x}^{2}+\vartheta }}, \end{array}$$

(4) $$\begin{array}{c} w_{x}^{2}=\frac{1}{e}\overset{a}{\underset{l=1}{\sum }}\left(s_{l}-w_{x}\right). \end{array}$$

In the above equation, equation (3) is the average value of batch size *q*, and equation (4) is the variance of batch size *q*.

When nonlinear factors are added to the ReLU layer, the expression ability of the increased model will be weakened. The activation function of ReLU is as follows:

(5) $$\begin{array}{c} f\left(m\right)=\max\left\{0,m\right\}. \end{array}$$

The main difference between the adaptive maximum pooling layer and the standard Max Pooling is that the former will control the output size (Out) according to the input size (In), and stride and kernel size are as follows:

(6) $$\begin{array}{c} \text{stride}=\text{floor}\left(\frac{\text{In}}{\text{Out}}\right),\\ \text{kernel size}=\text{In}-\left(\text{Out}-1\right)\times \text{stride},\\ \text{Padding}=0. \end{array}$$

The fully connected layer can be regarded as the full-scale convolution of *s* × *u*; *s* and *u* are the output size of the previous layer, and finally, 1026-dimensional features extracted by the convolutional neural network can be obtained:

(7) $$\begin{array}{c} h=\left(h_{1},h_{2},h_{3},\ldots ,h_{1026}\right). \end{array}$$

#### 2.4.2. Multimodal Feature Adaptive Fusion

Due to the different features of different modalities [16], a deep learning model of multimodal feature fusion is constructed to retain the correlation of multimodality. The model contains a hidden layer with a number of neurons less than the feature dimension and a Sigmoid layer. The entire network is trained by maximizing the energy proportion of the feature layer. The Sigmoid layer can map the feature interval after feature fusion to (0, 1), which is the prediction probability. The feature vector *m* = (*c*, *o*), and the forward propagation equation is as follows:

(8) $$\begin{array}{c} p_{e}=\left(s_{i}+t_{i}\right)\vartheta_{ie}+\beta_{e}, \end{array}$$

(9) $$\begin{array}{c} W=\partial \left(\sum_{l=1}^{a}\left(s_{i}+t_{i}\right)\vartheta_{ie}+\beta_{e}\right). \end{array}$$

In the above equations, ∂(*k*)=1/1+*n*^−*k*^, *t*_*i*_ is the deviation of the visible layer, *β*_*e*_ is the deviation of the hidden layer, and *p*_*e*_ is the hidden layer vector. To obtain the optimal fitting multimodal feature, the energy model is used to adjust the parameters, and the energy function is as follows:

(10) $$\begin{array}{c} H\left(x,y|\ell \right)=-\sum_{l=1}^{a}s_{i}t_{i}-\sum_{e=1}^{i}\beta_{e}p_{e}-\sum_{l=1}^{a}\sum_{e=1}^{i}t_{i}\vartheta_{ie}y_{i}. \end{array}$$

In equation (9), *ℓ*=(*t*_*i*_, *ϑ*_*ie*_, *y*_*i*_), *H*(*x*, *y|ℓ*) represents the total energy of the module.

The marginal probability distribution is defined as follows:

(11) $$\begin{array}{c} p\left(x|\ell \right)=\frac{1}{Z\left(\ell \right)}\sum_{e}r^{-k\left(x,y|\ell \right)}, \end{array}$$

(12) $$\begin{array}{c} p\left(y|\ell \right)=\frac{1}{Z\left(\ell \right)}\sum_{i}r^{-k\left(x,y|\ell \right)}. \end{array}$$

In equations (10) and (11), $Z\left(\ell \right)=\underset{il}{\sum }r^{-k\left(x,y|\ell \right)}$, and the optimization function is defined as follows:

(13) $$\begin{array}{c} \ell_{nm}=\underset{\ell }{\arg\;\max}\sum_{j=1}^{o}\mathrm{lg}P\left(x_{j}|\ell \right). \end{array}$$

In equation (12), *o* is the number of samples. When the function *ℓ* takes the maximum value, the energy proportion of the characteristic layer is high, and the energy of the hidden layer is small. When data is transmitted within the network, the direction of the data flow is also the direction of energy dissipation. After many iterations, the network energy shows a decay trend, the network tends to be ordered, or the probability distribution tends to be concentrated.

### 2.5. Evaluation Index

The performances of different models were quantitatively evaluated regarding the Accuracy, Recall, and AUC.

Accuracy refers to the proportion of the correct samples predicted by the model to the total samples, which is calculated as follows:

(14) $$\begin{array}{c} \text{Accuracy}=\frac{\text{TP}+\text{TN}}{\text{TP}+\text{FN}+\text{TN}+\text{FP}},\\ \text{Recall}=\frac{\text{TP}}{\text{TP}+\text{FN}}. \end{array}$$

In the above equations, TP (true positive) means that the segmentation result and the gold standard result are both true, that is, true positive. FP (false positive) means that the segmentation result is false, and the gold standard results are all true. FN (false negative)) indicates that the segmentation result is true, and the gold standard results are all false.

The AUC value is defined as the area under the ROC curve enclosed by the coordinate axis. Since the ROC curve is generally above the line *y* = *x*, the value range of AUC is between 0.5 and 1. The closer the AUC is to 1.0, the higher the authenticity of the detection method is.

The observation of concomitant injury of ACL mainly included common combined injuries such as meniscus tear, bone contusion, medial and lateral collateral ligament injury, cartilage injury, and joint effusion.

### 2.6. Statistical Methods

SPSS 19.0 was employed for data statistics and analysis. Mean ± standard deviation ($\bar{x}$ ± *s*) was how measurement data were expressed, and the comparison of the mean between each group was performed by *t* test. Percentage (%) was how count data were expressed, and the *χ*^2^ test was used. The difference was statistically considerable with *P* < 0.05.

## 3. Results

### 3.1. Analysis of the Results of ACL Damage Diagnosis Based on Deep Learning Algorithms

The results of ACL damage diagnosis based on deep learning algorithms were analyzed.  Figure 1 showed that, after fusion of traditional features and deep learning features, the performance indicators of MRI were improved to a certain extent, especially in accuracy and AUC value. The accuracy was up to 90%, and the highest AUC value was 0.9726. The detection rate of this model for general positive samples was higher than 92%, and the detection rate for positive samples of ACL tear and meniscus tear was high, which was of great significance to assist physicians in diagnosing high-risk patients.

From the results in Figure 1, the sagittal plane detection had a great advantage and a high accuracy of 96.28% in the task of ACL tear prediction. The prediction accuracy of meniscus tear was low, which was 75.37% (Figure 1(a)). In the prediction of recall rate, the prediction of ACL tear was the best on the horizontal axis, the recall rate was 89.56% (Figure 1(b)), and the AUC value was 0.9726. In the prediction of meniscus tear, the sagittal plane was the best, with a recall rate of 90.57% and an AUC value of 0.923 (Figure 1(c)).

Since each prediction task had only two cases of positive and negative, the prediction probability of the model greater than or equal to 0.5 was deemed as a positive patient, and the prediction probability less than 0.5 was deemed as a negative patient, so as to better show the prediction effect of the model. The test results of ACL tear and meniscus tear were shown in Figure 2. The results showed that this prediction model had good performance for ACL tear and meniscus tear predictions, especially for ACL prediction accuracy and recall rate, and the maximum AUC value was above 0.96. It indicated that the prediction model based on deep learning used in this study can be used as a basis for diagnosing knee joint injuries and had certain value in clinical adoptions.

### 3.2. MRI Features of Patients with Knee Joint Injury Based on Deep Learning

Figure 3 was the schematic diagram of a 55-year-old male patient with bone contusion (axial displacement sign). In Figure 3(a), once the ACL was torn, the tibia would move forward relative to the femur, causing the lateral femoral condyle to collide with the outer and posterior tibia. Both sides had edema, and the degree of knee flexion determined the location of the femoral condyle. Figures 3(b) and 3(c) were images of ACL tears observed at different positions.

Figure 4 showed MRI images of some patients with knee injuries.  Figure 4(a) showed ligament discontinuity. There was a low signal of the ligament, but the interruption was discontinuous, the path was low and flat, and the ligament was curled in a clumpy or wavy shape, which was generally seen in fresh injuries. In Figure 4(b), there was abnormal direction of ligament injury (ACL ptosis). There was a relatively intact ligament with low signal, but the direction was abnormal and pendulous, which was usually seen in the old injury of the femoral attachment, where the damaged ACL dropped and adhered to the PCL. In Figure 4(c), the ACL was absent. The intercondylar fossa was empty and there was no ligament signal. The symptoms were mainly present in prolonged injuries, where the damaged ACL tear was heavy and horse-tailed, did not enclose synovium, and was gradually corroded by enzymes in the joint.

In Figure 5(a), MRI T2WI showed a tear in the posterior horn of the medial meniscus of the knee. In Figure 5(b), MRI T2WI plain scan showed the high signal shadow within the low signal of the posterior cruciate ligament. The arrow indicated a partial rupture with hyperintensity bleeding around the rupture. The MRI diagnosis was an incomplete rupture of the right posterior cruciate ligament.

### 3.3. MRI Manifestations of ACL Injury

There are 60 knee joints in 30 patients with knee joint injury. In the examination results, the MRI examination showed that there were 34 cases of ACL grade III injury, 10 cases of grade II injury, 10 cases of grade I injury, and 6 cases of grade 0 injury. Arthroscopy showed that there were 34 cases of ACL grade III injury, 13 cases of grade II injury, 11 cases of grade I injury, and 2 cases of grade 0 injury. Compared with the results of arthroscopy, 3 cases were misdiagnosed as intact ligaments, 3 cases were misdiagnosed as grade II ligament injuries, 1 case was misdiagnosed as grade I ligament injuries, 4 cases were misdiagnosed as grade 0 injuries, and 2 cases were missed (Figure 6).

Figure 7 showed that the sensitivity, specificity, and accuracy of MRI in the diagnosis of ACL injury was 96.78%, 90.62%, and 92.17%, respectively, with no substantial difference from the results of arthroscopy (*P* < 0.05), which showed that MRI can accurately diagnose ACL injury.

### 3.4. ACL Injury Classification and Concomitant Injury

In this research project, there were 34 cases of ACL grade III injury, including 10 cases of chronic injury and 24 cases of acute injury, 10 cases of grade II injury, 4 cases of chronic injury, and 6 cases of acute injury. Among grade I and grade 0 injuries, chronic injuries accounted for 3 cases and acute injuries accounted for 13 cases. There were 43 cases of acute injury and 17 cases of chronic injury.

Among the types of ACL injuries, there were meniscus tears, bone contusions, internal and external collateral ligament injuries, cartilage injuries, joint effusions, etc. The common concomitant injury was the torn meniscus. There were 30 patients with acute injury in concomitant injury and meniscus injury. In addition, there were 20 patients with internal collateral ligament injury, 13 patients with lateral collateral ligament injury, 15 patients with cartilage injury, and 10 patients with bone contusion. Among chronic ACL injuries, 12 patients were accompanied by meniscus tears. In addition, there were 7 patients with collateral ligament injury, 5 patients with lateral collateral ligament injury, 7 patients with cartilage injury, and 3 patients with bone contusion.  Figure 8 shows the positive rate of ACL concomitant injury. The positive rate of acute ACL patients with bone contusion and medial collateral ligament injury was considerably higher than that of the chronic patients. However, the incidence of ACL injury with meniscus tear and cartilage injury in the chronic group was substantially higher than that in the acute group, and there was a remarkable difference between the two (*P* < 0.05).

## 4. Discussion

The main function of the ACL is limiting the overdevelopment of the tibial plateau and the rotation of the knee joint. During the bending movement of the knee joint, the fiber bundles in the knee joint obtain the stability of the knee joint through various stretching modes. When the knee joint is straightened, the posterolateral branch (PLB) is in tension, and the anteromedial branch (AMB) is slightly relaxed. When the knee joint is bent, AMB is in tension and PLB is in a relaxed state. When an external force acts on the knee joint, resulting in excessive extension or rotation (for example, excessive internal and external rotation), it is easy to cause ACL damage or even fracture. MRI has become the most ideal examination method for the diagnosis of knee cruciate ligament injuries due to its advantages of high contrast, high resolution, noninvasive, and multipart imaging. MRI can not only clearly show the normal form of ACL but also show the location, extent, fracture, tear of meniscus, and other knee joint injuries of injured ACL. In this work, a multimodal feature fusion model based on deep learning was proposed for imaging diagnosis based on MRI. First, the knee joint MRI image was preprocessed, and the multimodal features of knee joint injury were extracted based on both traditional and deep learning. Then, the multilayer neural network was adopted to perform correlation fusion of the features. The results showed that the sagittal plane detection has a great advantage and a high accuracy rate of 96.28% in the task of ACL tear prediction. The prediction accuracy of meniscus tear was low, which was 75.37%. In the prediction of recall rate, the prediction of ACL tear was the best on the horizontal axis, the recall rate was 89.56%, and the AUC value was 0.9726. In the prediction of meniscus tear, the sagittal plane was the best, with a recall rate of 90.57% and an AUC value of 0.923. This prediction model showed good prediction performance for ACL tear and meniscus tear. In particular, the prediction accuracy and recall rate of ACL were relatively better, and the maximum AUC value was above 0.96. The results were similar to the conclusions of Miyaji et al. [17] and both showed that the prediction model based on deep learning used in this study can be used as a basis for diagnosing knee joint injuries and had certain value in clinical applications.

The model was applied to the MRI diagnosis of ACL injury. The MRI examination results showed that there were 34 cases of ACL grade III injury, 10 cases of grade II injury, 10 cases of grade I injury, and 6 cases of grade 0 injury. Arthroscopy showed that there were 34 cases of ACL grade III injury, 13 cases of grade II injury, 11 cases of grade I injury, and 2 cases of grade 0 injury. Compared with the results of arthroscopy, 3 cases were misdiagnosed as intact ligaments, 3 cases were misdiagnosed as grade II ligament injuries, 1 case was misdiagnosed as grade I ligament injuries, 4 cases were misdiagnosed as grade 0 injuries, and 2 cases were missed. The sensitivity, specificity, and accuracy of MRI in the diagnosis of ACL injury was 96.78%, 90.62%, and 92.17%, respectively, and there was no great difference from the results of arthroscopy (*P* > 0.05). Namiri et al. [18] found that the indirect signs of ACL tear had high specificity (91%∼100%) and sensitivity in a retrospective study of the correlation between MRI imaging and arthroscopy in 100 patients. Therefore, these signs can determine whether the patient had an ACL tear, which was similar to the conclusion of this study, indicating that MRI can accurately diagnose ACL injury. The positive rate of acute ACL patients with bone contusion and medial collateral ligament injury was notably superior to the chronic group. However, the incidence of ACL injury with meniscus tear and cartilage injury in the chronic group was substantially higher than that in the acute group, with substantial differences (*P* < 0.05). Pedoia et al. [19] reported a high incidence of combined articular cartilage damage. However, the literature did not separate statistics on acute and chronic injuries. In this research topic, a clear analysis of the types of concomitant damage was carried out, and the results also provided a certain reference for the diagnosis of ACL concomitant damage.

## 5. Conclusion

A multimodal feature fusion deep learning model based on deep learning algorithms was established in this work and applied to the diagnosis of ACL injury patients, to explore the value of MRI based on deep learning in the diagnosis of ACL injury. The results revealed that deep learning-based MRI substantially improved the ability to diagnose ACL damage and increased the sensitivity, specificity, and accuracy of the diagnosis of ligament damage. However, this study still has some shortcomings. The number of patient samples selected is small, there is a lack of disease diversity research, and the scope of adoption of the research results has certain limitations. In the future work, the research area and research samples will be further expanded to ensure the universality of research results. In summary, the ability to diagnose ACL injuries in MRI images based on deep learning is improved, which provides a reference for the diagnosis and treatment of patients with knee joint injuries.

## Figures and Tables

**Figure 1:** Analysis of diagnosis results of ACL injury based on deep learning algorithm. Accuracy comparison of transverse plane, coronal plane, and sagittal plane (a); recall rate comparison of transverse plane, coronal plane, and sagittal plane (b); AUC comparison of transverse plane, coronal plane, and sagittal plane (c). ^*∗*^indicated that the accuracy, recall rate, and AUC of ACL injury were statistically different from that of meniscus injury (*P* < 0.05).

**Figure 2:** Performance comparison of regression models: (a) comparison of accuracy and recall rate of ACL and meniscus tear; (b) comparison of AUC of ACL and meniscus tear. ^*∗*^indicated that ACL injury was dramatically different versus meniscus injury (*P* < 0.05).

**Figure 3:** Schematic diagram of ACL injury. (a) The ACL tear, the arrow indicated the site of the ligament injury, (b) the coronal diagram of the ligament tear, and (c) the sagittal diagram of the ligament tear.

**Figure 4:** MRI images of the patients. (a) ACL discontinuity (49-year-old female patient), (b) ACL drooping sign (58-year-old male patient), and (c) ACL disappearance (55-year-old male patient).

**Figure 5:** MRI T2WI images of the patients (male, 61 years old). (a) Tear of posterior corner of medial meniscus of knee joint (the arrow was the tear site); (b) MRI T2WI plain scan of posterior cruciate ligament (the arrow indicated a partial rupture of the ligament).

**Figure 6:** MRI diagnosis result of ACL injury.

**Figure 7:** Contrast of MRI diagnosis performance of ACL injury.

**Figure 8:** Contrast of positive rate of ACL concomitant injuries (A: bone contusion; B: medial collateral ligament injury; C: meniscus tear; D: cartilage injury; E: lateral collateral ligament injury) (^*∗*^suggested remarkable differences in contrast to acute injury, *P* < 0.05).

## Data Availability

No data were used to support this study.
